# Rehardening of Eroded Enamel with CPP-ACFP Paste and CO_2_ Laser Treatment

**DOI:** 10.1155/2021/3304553

**Published:** 2021-07-14

**Authors:** Shahin Kasraei, Parmis Kasraei, Sara Valizadeh, Mohadeseh Azarsina

**Affiliations:** ^1^Department of Restorative Dentistry, Dental School, Shahid Beheshti University of Medical Sciences, Tehran, Iran; ^2^Roshangaran High School, District 3, Tehran, Iran; ^3^Dental Research Center, Dentistry Research Institute, Restorative Dentistry Department, Dental School, Tehran University of Medical Sciences, Tehran, Iran; ^4^Department of Operative Dentistry, Dental School, Shahid Beheshti University of Medical Sciences, Tehran, Iran

## Abstract

**Background:**

Diet and lifestyle can destroy tooth structure due to the dissolution of enamel by acidic beverages. The present study evaluated the effect of CO_2_ laser irradiation and CPP-ACFP (casein phosphopeptide and amorphous calcium phosphate with fluoride) paste on the remineralization of enamel eroded by carbonated soft drinks.

**Methods:**

In the present in vitro study, 46 human sound premolar teeth were sectioned mesiodistally to achieve 84 samples. Fourteen samples were assigned to the positive control group (G1), and the remaining samples were immersed in 500 mL of cola drink for 2 minutes, followed by rinsing with distilled water for 10 seconds. This procedure was carried out three times to create erosive lesions. Then, the 60 eroded samples were randomly assigned to five groups of G2 to G6 in terms of the treatment as follows: negative control (G2), CO_2_ laser irradiation (G3), CPP-ACFP paste (G4), CO_2_ laser irradiation followed by CPP-ACFP paste application (G5), and CPP-ACFP paste application followed by CO_2_ laser irradiation (G6). The mean surface microhardness of the enamel surface was evaluated and determined at three points for each sample. Data were analyzed with one-way ANOVA and Tukey HSD tests (*α* = 0.05).

**Results:**

The highest and the lowest hardness values were recorded in the G1 (314 ± 12 kg/mm^2^) and G2 (213.7 ± 12 kg/mm^2^) groups, respectively. ANOVA revealed significant differences between the study groups (*P* < 0.001). Two-by-two comparisons showed significant differences between the G2 group and the other groups, indicating the efficacy of all the treatment modalities in tooth remineralization and rehardening procedures (*P* < 0.05). Only in group G6, the enamel microhardness was not significantly different from the G1 positive control group (*P* > 0.05).

**Conclusion:**

Considering the parameters used in the present study, CO_2_ laser irradiation or CPP-ACFP paste application alone increased eroded enamel's surface hardness; however, their sequential application was more effective in rehardening the eroded enamel's surface to near-normal levels.

## 1. Introduction

The teeth undergo continuous demineralization and remineralization in the oral cavity; these two processes should generally be balanced. However, when demineralization becomes dominant in the oral cavity conditions, progressive destruction of the enamel surface occurs [1].

The most critical factor for tooth demineralization is the acid produced by cariogenic bacteria. Dental caries is the second most common infectious disease after respiratory diseases [2]. Besides, the loss of enamel inorganic structure might occur due to erosive processes. One of the most critical risk factors for tooth erosion is excessive consumption of soft drinks with erosive properties that decrease salivary function and compromise the enamel structure [3]. Low-pH soft drinks, including fresh citrus fruit juice, carbonated acidic drinks, and sports supplemental drinks, can cause tooth erosion. Tooth erosion incidence has increased due to an increase in the consumption of acidic soft drinks in recent years. In the past 20 years, a lifestyle change has increased the American adult population's consumption of acidic soft drinks by 300% [4]. Besides, the alimentary tract acid and conditions related to digestive tract dysfunction, including reflux, anorexia nervosa, and bulimia, are some risk factors for tooth erosion. In addition to identifying the etiologic factors for these lesions, it is important to diagnose these conditions early and render preventive treatment [5].

The inorganic contents of tooth hard structures are lost due to the exposure to acid with a bacterial and nonbacterial origin, decreasing tooth hardness [6]. The tooth hard tissue loss is due to two important processes: (1) dissolution of enamel's apatite crystals; (2) diffusion of calcium, phosphate, and hydrogen ions into and out of the enamel microstructures. Tooth enamel demineralization is a dynamic process that beings with the formation of incipient subsurface lesions. If the demineralization process continues, incipient clinical lesions will result in enamel cavitation [7].

The remineralization of decalcified enamel and restoration of its surface hardness are two important and challenging aims in dentistry. Despite some old techniques, including regular dental visits and toothbrushing with fluoridated toothpaste, more effective interventions are necessary in some cases [8–10]. It has been demonstrated that the enamel demineralization and remineralization depend on the acidity and the concentration of ions in the aqueous environment surrounding the tooth structure [11].

Currently, several clinical methods, including fluoride therapy, the use of CPP-ACP (casein phosphopeptide–amorphous calcium phosphate), laser irradiation, or a combination of laser and remineralizing agents, are suggested to increase tooth resistance against the loss of its hard structures [10–12].

Since calcium, phosphorus, and fluoride ions have a critical role in enamel remineralization, topical use of some materials, such as CPP-ACP paste or fluoride-containing materials, has been considered to increase tooth resistance to prevent or treat enamel demineralization [13, 14]. It has been reported that when fluoride is incorporated into CPP-ACP paste, it will have a synergistic effect on the enamel remineralization process [12].

The application of laser technology has been reported to decrease hydroxyapatite crystals' solubility in acidic environments with proper wavelengths of laser beams on the enamel surface [15–17]. The CO_2_ laser with a 10.6 *μ*m wavelength induces chemical and morphological changes in the enamel structure, changing its mineral and organic content and incasing its resistance against acid attack and caries [17, 18].

To the best of our knowledge, the effect of the combined use of laser beams and CPP-ACFP paste or their sequential use on eroded enamel remineralization and rehardening has not been adequately studied. Therefore, the present study is aimed at evaluating the effect of CO_2_ laser beams with or without CPP-ACFP paste on restoring eroded enamel surface hardness.

The null hypothesis was that CO_2_ laser irradiation and treatment with CPP-ACFP paste do not affect the surface hardness of eroded enamel.

## 2. Materials and Methods

This in vitro study with protocol number p16/9509235539 was approved by the ethics committee of the dental school.

Forty-two sound human premolar teeth extracted for orthodontic reasons were collected and cleaned with a scalpel blade and a toothbrush, followed by storage in normal saline solution at room temperature. The teeth were disinfected with 0.5% chloramine T solution one week before undertaking the study. The coronal surfaces of the teeth were evaluated under a stereomicroscope to ensure the absence of structural defects, cracks, and caries. Each tooth crown was removed at CEJ using a diamond disk under water cooling. Then, each tooth crown was divided into facial and palatal halves.

The prepared samples were mounted in self-cured acrylic resin (Acropars, Kaveh, Tehran, Iran), with a 4 × 4 mm area of the smoothest facial or palatal enamel surface exposed. The sample surfaces were abraded with wet 600- and 1200-grit abrasive paper in association with water to achieve a smooth and finished enamel surface. The samples were stored in distilled water to prevent dehydration. Fourteen enamel samples were assigned to the positive control group with no surface treatment (G1), and the remaining samples were immersed in nonalcoholic carbonated cola drink (Coca-Cola, Mashhad, Iran) for 2 minutes to erode the enamel surface, followed by rinsing with distilled water for 10 seconds. The procedure was repeated three times, and each time, a fresh cola drink was used; therefore, the samples were immersed in the erosive cola drink for 8 minutes in total. The drink's pH was determined at 20°C (pH = 2.5) with a pH meter (Metrohm 744, Herisau, Switzerland). Then, the eroded samples were randomly assigned to five groups (*n* = 14), as follows:

G2: the eroded samples did not undergo any treatment (negative control).

G3: the samples were only irradiated with CO_2_ laser beams.

G4: the eroded samples were treated only with a commercial paste of CPP-APFC.

G5: the eroded samples were first irradiated by CO_2_ laser beams and then treated with CPP-APFC paste.

G6: the eroded samples were first treated by CPP-APFC paste and then irradiated with CO_2_ laser beams.

After the interventions, the samples were immersed in artificial saliva (pH = 7.0) for 48 hours.

The CPP-ACFP (MI Paste Plus, Recaldent™, GC Co., USA) paste was applied to the eroded enamel surface in the form of a circle measuring 3 mm in diameter and 1 mm in thickness for three minutes with a swab according to the manufacturers' instructions and then rinsed with water for 10 minutes.

CO_2_ laser beams were applied with a 10.6 *μ*m wavelength to lase the enamel surface using the following parameters: power of 0.7 W, pulse duration of 0.4 milliseconds, a spot size of 0.4 mm, pulse frequency of 50 Hz, and focal spot of 0.2 mm. CO_2_ laser beams were irradiated with the hollow tube tip from a 10 mm distance to the enamel surface in noncontact mode. The applied laser fluence was 10.66 J/cm^2^, and the average power output was 0.68 W, which was measured by using a laser power meter (Model 37-3002, Scientech Inc, Colorado, USA). During the CO_2_ laser beam irradiation on the samples, air spray was blown at 60% to the lased surface. The enamel surface was uniformly scanned with a circular movement in a circle measuring 3 mm in diameter at a speed of 2 mm/s in an outward direction for 10 seconds.  Figure 1 shows laser setting and materials used in this study.

After the treatment procedures, all the samples were immersed in artificial saliva for 48 hours, consisting of 0.7 mmol/L of CaCl_2_, 0.2 mmol/L of MgCl_2_·6H_2_O, 4 mmol/lit of KH_2_PO_4_, 30 mmol/lit of KCl, and 20 mmol/L of HEPES buffer (pH = 7).

In the final step, a Knoop surface hardness tester (Zcwik-Roell, Germany) was used to determine the enamel surface microhardness in the central area of all the samples with a 25 g force with a dwell time of 10 seconds at three points, at least 300 *μ*m apart from each other. The means of the three measurements were calculated and recorded as the Knoop hardness number (KHN) of the samples in kg/mm^2^ [19].

The data were analyzed with SPSS using one-way ANOVA and post hoc Tukey tests at a significance level of *P* < 0.05.

## 3. Results

The means and standard deviations of surface hardness of the study groups are presented in Table 1. The highest surface hardness was recorded in the positive control group (G1) (314 ± 12 kg/mm^2^), and the lowest was recorded in the negative control group (G2) (213 ± 12 kg/mm^2^). One-way ANOVA showed significant differences between the study groups (*P* < 0.001).

Two-by-two comparisons of the groups with post hoc Tukey tests showed that the means of surface hardness of all the groups were significantly higher than the negative control group (*P* < 0.05). Besides, the mean surface hardness of groups G3, G4, and G5 was not significantly different (*P* > 0.05). Furthermore, the results showed that the mean surface hardness of only group G6 (307.57 ± 20 kg/mm^2^), in which the CPP-ACFP paste was applied, followed by CO_2_ laser beam irradiation sequentially, was not significantly different from the positive control group (314 ± 12 kg/mm^2^), in which no treatment was applied (*P* > 0.05).

## 4. Discussion

Nowadays, the treatment of enamel erosive lesions and incipient caries has become an important challenge in dentistry due to the increased consumption of carbonated soft and energy drinks. Different techniques have been suggested to prevent and treat these lesions, including the use of fluoride and mineralizing agents and different surface preparation techniques, including laser beams [15, 20].

Different techniques are used to determine the severity of enamel demineralization, including QLF, polarized light microscopy, and micrographs. Since microhardness is correlated with the mineral content of teeth, enamel surface hardness determination is one of the valuable, indirect, and reproducible techniques used to evaluate enamel remineralization in in vitro studies [1, 20]. Therefore, enamel surface hardness was determined to evaluate the effect of CO_2_ laser irradiation and CPP-ACFP paste on the remineralization of enamel eroded by carbonated soft drinks in the present study.

In the present study, group G2 (213.7 ± 12 kg/mm^2^) exhibited a significant decrease in enamel surface microhardness compared to group G1 (314.0 ± 12 kg/mm^2^), in which no treatment was carried out, indicating the effect of carbonated soft drinks on the induction of erosive lesions and enamel demineralization. In all the study groups, except for group G2, there was a significant increase in the surface hardness of demineralized enamel after a therapeutic intervention with CO_2_ laser and CPP-ACFP paste, consistent with some previous studies [13, 17, 18, 20, 21].

CPP-ACP is prepared by precipitating calcium and phosphorus on casein, a digestible milk protein [13]. Casein phosphopeptides are adhesive proteins that bind to calcium and phosphate ions and are stabilized in an amorphous state. This complex adheres to the salivary pellicle, plaque, and soft tissues, and even hydroxyapatite components. CPP has a vital role as a carrier for ACP in concentrating the soluble phases of calcium and phosphate on the tooth surface. CPP binds to calcium and phosphate through the phosphoserine in its structure and forms small ACP clusters on the tooth surface. These nanocomplexes (pH = 5.9) increase tooth remineralization [20]. The CPP-ACP paste preserves mineral agents' saturation, especially calcium and phosphate, on the tooth surface, inhibiting cariogenic agents' activity and increasing remineralization [14, 18, 20, 22, 23]. A 10-year systematic review showed that CPP-ACFP had a much significant effect than placebo on tooth remineralization, and the effect of this paste depended on its type and its frequency and duration of application [15]. In some studies, the application of CPP-ACP paste increased the surface hardness of demineralized enamel even more than the sound samples, which was attributed to the supersaturated metastable calcium and phosphate solution [23]. Esfahani et al. showed that fluoride in the CPP-ACP structure significantly increased the remineralization effect and the salivary buffering capacity. The incorporation of fluoride into CPP-ACP paste and the fluoride ions in its structure increased its effect on enamel remineralization compared to CPP-ACP and fluoride varnish alone [24].

Some previous studies have shown that the efficacy of therapeutic interventions with materials containing fluoride, calcium, and phosphorus is higher than that of laser irradiation alone, and laser irradiation of the enamel alone cannot prevent caries [25], consistent with the present study. However, the report that laser irradiation alone did not increase enamel surface hardness or simultaneous use of these two techniques did not significantly increase enamel surface hardness is contrary to the present study results, which might be attributed to differences in the laser or the sequence of the use of remineralizing agents and laser irradiation.

The application of CO_2_ laser beams to the enamel surface increased enamel remineralization to some extent, and the numeric value of surface hardness increased significantly compared to the negative control group (G2). However, this amount of increase in enamel surface hardness in the group in which only CO_2_ laser beams were used was less than that in the other study groups.

CO_2_ laser with 9.3, 9.6, 10.3, and 10.6 *μ*m wavelengths should rank first to prevent enamel erosion and caries among all the other lasers that are used in dentistry for preventive purposes because the wavelength bands that are absorbed by phosphate, carbonate, and hydroxyl ions in the enamel and dentin structure are in the 9–11 *μ*m range, consistent with CO_2_ laser beam wavelengths [15, 26]. After the absorption of laser beams, there is a significant increase in the surface and subsurface layers' temperature, resulting in chemical and structural changes in enamel, including decreased carbonate ions, fusion, and recrystallization of hydroxyapatite crystals, which make the tooth surface more acid-resistant [27]. By considering a proper fluence of the irradiated laser energy to the enamel surface, the CO_2_ laser with a 10.6 *μ*m wavelength is more effective in increasing resistance to acid than its 9.6 *μ*m wavelength due to its lower absorption coefficient and deeper enamel penetration. It has been demonstrated that CO_2_ laser irradiation with specific wavelengths decreases demineralization up to 98% and resistance to acid attack up to a depth of 58 *μ*m [3]. Esteves-Oliveira et al. reported that CO_2_ laser beams could reharden the acid-softened enamel [28]. CO_2_ laser beams can melt dentin, occluding dentinal tubules. Besides, the heat produced by laser beams is associated with the release of water, organic components, and carbonate ions that have a weak bond and high solubility from the hydroxyapatite structure. These laser beams form the tetracalcium diphosphate monoxide crystalline phase at 650–1000°C, which is more resistant to demineralization [29].

Some studies have shown the adverse and decreasing effects of laser beams on enamel surface hardness [30, 31]. The application of high-power laser beams with inappropriate parameters can lead to irregularities and cracks on the tooth surface, increasing enamel surface brittleness and decreasing its surface hardness, which serves as points for the initiation of acid attacks [30]. It should be emphasized that CO_2_ laser beams with subablative parameters change the chemical composition and morphology of dental substrate and increase its resistance to acid attack by decreasing its penetrability and solubility and denaturing the remaining organic matrix [32]. A study by Kuramoto et al. showed that if the enamel is irradiated with a low-level laser (i.e., 3–21 j), hardness will increase to some extent, but if the enamel is irradiated with a high-energy level (i.e., 30–100 j), the surface hardness will decrease [33]. Laser beams with high power and energy cause enamel cracks, resulting in a decrease in surface hardness. However, if appropriate laser beam parameters are selected, they can induce favorable changes in the enamel structure to increase its resistance to acid attack and demineralization. Rodrigues et al. showed that CO_2_ laser increased resistance to demineralization in enamel, which further increased with fluoride use [34]. They reported that laser beams were more effective than fluoride in preventing caries, in contrast to the present study, which might be attributed to the use of toothpaste as a fluoride source with a lower fluoride content than the material used in the present study.

The present study showed that the concomitant and sequential use of CPP-ACFP and CO_2_ laser beams (group G6) had the most significant effect on restoring the surface hardness of acid eroded enamel to the level of sound enamel. Therefore, if there is a time limitation for the repeated application of enamel remineralizing agents, or in children or cases where there are concerns about the use of high fluoride concentrations, the simultaneous use of enamel remineralizing agents and sequential laser irradiation might be a proper choice for treating erosion and preventing caries.

Concerning the effect of these two methods combined, there are contradictory opinions about laser beams' impactions before, during, or after using remineralizing agents and fluoride to prevent caries and treat eroded enamel [3, 16, 30]. Some studies have shown that the use of CPP-ACFP and CO_2_ laser increases tooth microhardness through a synergistic effect, consistent with the present study [30, 31]. Different reasons have been suggested to explain this synergistic effect. It has been reported that during the melting and rehardening process of the tooth structure by laser beams, globular granules form on the enamel surface, and when supersaturated calcium, phosphate, and fluoride ions are present on the enamel surface, the chances of these ions' penetration into the microscopic intergranular spaces and their precipitation on the enamel subsurface layer increase, therefore were caused decreasing enamel penetrability [34]. Besides, during recrystallization in the guided presence of ACP by CPP, larger and more organized crystals of HA are formed, increasing enamel hardness [16].

Dionysopoulos et al. reported that the laser's thermal effect creates different surface cracks, where minerals and fluoride are trapped, and finally converting loose surface minerals into firmly bonded minerals [14]. Besides, laser irradiation can increase the adhesion and bonding of fluoride to the tooth structure, leading to a higher fluoride content in contact with the enamel. In addition, the apatite produced in an environment containing calcium and phosphorus has a lower carbonate and manganese content, making it more resistant to acid attacks. The penetration and adhesion of calcium and phosphate nanoclusters to the enamel surface serve as reservoirs for ions, which help enamel remineralization by replacing ions in the subsurface layers [35].

However, in studies by Heravi et al. [16] and Asl-Aminabadi et al. [23], such a synergistic effect was not observed, which might be due to different lasers (Er: YAG and Nd: YAG) or different laser parameters used in those studies. Also, the substrate used in the studies above was deciduous tooth enamel, which is different in its structural properties, caries induction, and erosion from the permanent tooth enamel.

As shown in the present study, the sequence of the application of CPP-ACFP paste and subsequent CO_2_ laser beams might affect the treatment outcomes and the increase in enamel surface hardness (Table 1). Therefore, the sequence of using remineralizing agents and laser irradiation should be considered in the combined protocol of enamel surface rehardening. It has been demonstrated that an increase in enamel surface temperature up to 300–400°C due to laser irradiation increases enamel's resistance to demineralization; however, it decreases ion diffusion and penetrability of enamel [14]. It seems that the heat produced due to the fluence of energy from the irradiated laser beams increases the surface hardness and decreases enamel carbonates. On the other hand, they can decrease the diffusion of ions into prismatic and interprismatic spaces by denaturing the enamel organic matrix and decreasing interprismatic spaces, affectig the positive effects of CPP-ACFP paste [36].

The present study showed that the surface hardness of eroded enamel after the combined and sequential use of laser and CPP-ACFP are more effective than the laser or remineralizing pastes alone in rehardening enamel through the synergistic mechanisms mentioned above. However, if the remineralizing paste is used first, and after the ions' absorption to the surface or inside the enamel, the CO_2_ laser is applied with appropriate parameters, and a better rehardening effect of the enamel will be achieved.

It should be pointed out that in the present study, although all the collected teeth belonged to patients from a specific age group and the procedures were carried out by one operator, due to the *in vitro* design of the study and limitations such as the difficulty to simulate the oral conditions, with the same demineralization and remineralization cycles, the absence of salivary flow, oral bacteria, and other oral protective factors such as salivary proteins, further clinical studies are necessary, as concluded in previous studies [15, 37].

## 5. Conclusion

It can be concluded from the results of the present study that the use of CPP-ACFP followed by CO_2_ laser irradiation with proper parameters can significantly increase enamel surface hardness, and it is more effective than using these methods and materials alone for enamel remineralization.

## Figures and Tables

**Figure 1:** Laser setting and materials used in this study.

**Table 1:** Comparison of mean difference microhardness (kg/mm^2^) values of studied groups.

Groups	Mean ± SD	95% confidence interval for mean		Minimum	Maximum	^∗^ *P* value
		Lower bound	Upper bound			
(G1) Negative control	314.0 ± 12 A	306.6	321.3	294	337	0.0001
(G2) Positive control	213.7 ± 12 B	206.2	221.2	195	236	
(G3) CO_2_ laser	266.3 ± 21 C	254.1	278.5	235	306	
(G4) CPP-ACFP	270.7 ± 23 C	257.2	284.2	241	318	
(G5) Laser+CPP-ACFP	286.2 ± 26 C	271.0	301.5	251	331	
(G6) CPP-ACFP+laser	307.5 ± 20 A	295.4	319.6	269	339	

^∗^One way-ANOVA; same capital letters show no difference by using POH Tukey HSD tests (*P* > 0.05).

## Data Availability

All data are available if required.
